The article "Determinants and Trends of Health Facility Delivery in Bangladesh: A Hierarchical Modeling Approach" was published in 2022. Journal: Biomed Res Int.

# Determinants and Trends of Health Facility Delivery in Bangladesh: A Hierarchical Modeling Approach

**DOI:** 10.1155/2022/1359572

**Published:** 2022-07-29

**Authors:** Samia Kabir, Md. Rifat Hasan, Md. Ismail Hossain, Sharmin Suraiya, Fiza Binta Islam, Md. Iqbal Hossain Nayan, Iqramul Haq, Md. Sanwar Hossain

**Affiliations:** ^1^Department of Statistics, Jagannath University, Dhaka 1100, Bangladesh; ^2^Department of Pharmacy, East West University, Dhaka 1212, Bangladesh; ^3^Department of Agricultural Statistics, Sher-e-Bangla Agricultural University, Dhaka 1207, Bangladesh

## Abstract

**Background:**

Most maternal deaths occur during childbirth and after childbirth. This study was aimed at determining the trends of health facilities during delivery in Bangladesh, as well as their influencing factors.

**Methods:**

This study used secondary data from three Bangladesh Multiple Indicator Cluster Surveys (MICSs) in 2006, 2012–13, and 2019. The study's target sample was those women who gave birth in the last two years of the survey. A two-level logistic regression was applied to determine the effects on health facility delivery separately in these two survey points (MICSs 2012–13 and 2019).

**Results:**

The results show that the delivery of health facilities has increased by almost 37.4% in Bangladesh, from 16% in 2006 to 53.4% in 2019. The results of two-level logistic regression show that the total variation in health facility delivery across the community has decreased over recent years. After adding community variables, various individual-level factors such as women with secondary education (OR = 0.55 in 2012-13 vs. OR =0.60 in 2019), women from middle wealth status (OR = 0.49 in 2012-13 vs. OR = 0.65 in 2019), religion, and child ever born showed a strong relationship with health facility delivery in both survey years. At the community level, residents showed significant association only in the 2012-13 survey and indicated a 43% (OR = 1.43 for 2012-13) greater availability of health facilities in urban residences than in rural residences. Using media showed a highly significant connection with health facility delivery in both years as well as an increasing trend over the years in Bangladesh (OR = 1.19 in 2012-13 vs. OR = 1.38 in 2019). However, division, prenatal care, and skilled services all contribute greatly to increasing the delivery of health facilities in Bangladesh.

**Conclusions:**

The results of this study suggest that policymakers need to pay attention to individual and community-level factors, especially women's education, poverty reduction, and adequate prenatal care provided by well-trained caregivers.

## 1. Introduction

The global maternal mortality rate declined by 38% between 2000 and 2017 [1]. Meanwhile, coverage for health facilities during delivery has increased outstandingly across the globe. Although women's health well-being has improved throughout the world, it remains elusive in lower-middle-income areas such as sub-Saharan Africa and South Asia. The lack of awareness of health in developing countries such as Ghana is a significant challenge [2]. Bangladesh is one of the most populous developing countries with a poverty rate of 33% and various health problems [3, 4]. The country has established extensive health infrastructure in order to achieve the Sustainable Development Goals (SDGs) [5].

Healthy lifestyles are part of SDG 3 [6] by ensuring and promoting them for all people. Several other SDG goals are associated with this goal. As part of Sustainable Development Goal 3, the first goal is to reduce the global maternal mortality rate to less than 70 per thousand live births by 2030, to ensure that there is no alternative to upgrading the facility's health services.

Since most maternal deaths occur during pregnancy of childbirth, low- and middle-income countries are placing greater emphasis on facility delivery [7]. Facilities refer to institutional delivery, antenatal care (ANC), skilled birth attendants, etc., which reduce the risk of pregnancy-related complications for pregnant women. During pregnancy, antenatal care plays a crucial role in both the infant development and the overall health of the mother [8].

In many cases, maternal deaths are caused by obstetric conditions, including obstructed labor, hemorrhage, unsafe abortion, and hypertension disorders [9]. Consequently, women need antenatal care, an experienced medical birth attendant, a facility for healthy delivery, and postnatal care, all of which result in quality care. Even in extreme situations, quality care is possible [10]. However, only about 37% of Bangladeshi women deliver in a designated health facility [11], and this percentage will increase further if women are informed about prenatal health care. Several studies have also found that women are more likely to seek treatment in health facilities when they are told about pregnancy complications during antenatal care [12, 13]. The quality of obstetric and newborn care is another factor that can reduce maternal and newborn mortality [14]. Several studies in Bangladesh have identified some factors that influence health care. Place of residence [15–17], mother's age [16], division [17, 18], education of mother [15–17], parity [17, 19], availability of media [20], access to prenatal care [21], etc. are listed as important factors in the provision of healthcare.

In the past, several researchers have tried to determine the factors that affect whether a woman delivers in a health facility or not by using various techniques and different statistical models. In most studies, binary logistic regression models are most commonly used. Perkins et al. [22] and Ahinkorah et al. [23] attempted to uncover the determinants of the delivery of health facilities by using a binary logistic regression model but identified only individual factors. However, community factors also influence medical care. In several studies, community or social factors have already been shown to play a role in the utilization of maternal health services in South Asia and Africa. Studies conducted by Huda et al. in 2019 [16] and Olorunsaiye et al. in 2019 [24] in Bangladesh and Africa also attempted to identify the effect of community factors. However, in Bangladesh, people are less aware of the role of community factors in the use of health services. Based on this gap, this study tried to use data from three Bangladesh Multiple Indicator Cluster Surveys conducted in 2006, 2012-13, and 2019, and to explore the trend of using health facilities during delivery. This study used all two survey time points and determined the effects of factors (both individual and community). Only 2012-13 and 2019 Bangladesh MICSs data was used to fit a two-level model to determine individual and community care factors in Bangladesh.

## 2. Materials and Methods

### 2.1. Data Source

This study is based on secondary cross-sectional data and is nationally representative, named the Bangladesh Multiple Indicator Cluster Surveys (MICSs), which was managed by the Bangladesh Bureau of Statistics (BBS) and funded by UNICEF in Bangladesh. The study analysis was based on three Bangladesh MICSs conducted in 2006, 2012-13, and 2019. The data collection process for Bangladesh MICS, 2006 began in July and finished in December 2006, for Bangladesh MICS, 2012-13 began in December 2012 and finished in May 2013, and for Bangladesh MICS, 2019 began in January and finished in June 2019. The MICS used a two-stage stratified cluster sampling procedure to cover the population of Bangladesh's noninstitutional dwelling units. A more detailed description of the research environment, sampling methods, and data collection procedures can be found on the official MICS website, which is https://mics.unicef.org/.

MICS used four types of questionnaires for data collection purposes, namely,

1. household questionnaires
2. woman's questionnaires
3. man's questionnaires
4. children's questionnaires

The women's survey respondents aged 15-49 were used for the analysis. The Bangladesh MICSs covered 68247, 55120, and 64400 residential households from 2006, 2012-13, and 2019, respectively. Of these selected households, 78260, 51791, and 68709 women aged 15 to 49 years were qualified. The data weighted for this research purpose was provided by MICS authorities, and the final sample size for this study was 69860, 51791, and 64378 from 2006, 2012-13, and 2019, respectively. Case selection was restricted to the subset of women who gave birth in the preceding two years, so the sample size was considered to be 11899, 7950, and 9183 women between 15 and 49 years of age from 2006, 2012-13, and 2019, respectively. The complete process of sample design and sample selection is shown in Figure 1. This study has not been able to use the Bangladesh MICS, 2006 dataset in bivariate and multivariate analysis as many variables related to this study were missing. Therefore, Bangladesh Multiple Indicator Cluster Survey datasets for 2012-13 and 2019 were used to continue the bivariate and multivariate analysis in this study.

### 2.2. Outcome Variable

The binary outcome variable was facility delivery, which includes the location of delivery and is dichotomously classified as a “yes/no” variable. A birth was described as facility-based if it occurred in any public or private hospital, with all facilities classified as “yes,” otherwise as “no.”

### 2.3. Explanatory Variables

This study divided explanatory variables into two categories: individual-level factors and community-level factors. Women's age (in years) (15-19, 20-34, and 35-49) [25], women's education (preprimary/none, primary, secondary, and higher+) [25], wealth status (poor, middle, and rich) [26], religion (Islam and others) [27], wanted children (yes and no), and children ever born (1, 2-3, and >3) were considered individual factors for this study. This study considered the census enumeration cluster or block as a community. We include the residence type (urban and rural) as a proxy measure of community characteristics, division (Barishal, Chattogram, Dhaka, Khulna, Mymensingh, Rajshahi, Rangpur, and Sylhet), mass media exposure (exposure and not exposure), prenatal care (none, 1-3, and >3) [27], and skilled prenatal providers (yes and no) [28] as community-level factors. The wealth index is a composite indicator of wealth. MICS constructs the wealth index by applying the principal component analysis method, which is performed by using the information on the ownership of consumer goods, dwelling characteristics, water and sanitation, and other characteristics that are related to the wealth of the household. In terms of mass media, women aged 15 to 49 years who, at least once a week, read a newspaper or magazine, listen to the radio, and watch television, this study codes it as exposure, otherwise not exposure [28].

### 2.4. Analysis Procedure

This study performed a frequency distribution with percentages to present the summary of the explanatory variables. To explore the association between dependent and explanatory variables, a *χ*^2^ test was performed. Mathematically, the chi-square statistics can be defined as

(1) $$\begin{array}{c} \chi^{2}=\overset{n}{\underset{i=1}{\sum }}\frac{{\left(\text{Observed frequenc}{\text{y}}_{\text{i}}-\text{Expected frequenc}{\text{y}}_{\text{i}}\right)}^{2}}{\text{Expected frequenc}{\text{y}}_{\text{i}}}. \end{array}$$

This statistic follows a chi-square distribution with (Number of row − 1) × (Number of column − 1) degrees of freedom.

In a multivariate setting, random intercept multilevel logistic regression has been performed to analyze the effects of individual and community-level factors on the delivery of health facilities. The study used a multilevel modeling procedure for the hierarchical structure of data. The intraclass correlation coefficient (ICC) should be calculated before using any multilevel model. If the ICC value is greater than 0, a multilevel logistic regression model can be used [29]. In our survey, the individual was nested within the family, and the family was nested within the community.

First, we fitted an empty model (model 1) with a random intercept only. Then, the second model was fitted that included all individual factors (model 2). Finally, model 3 included both individual- and community-level factors as independent variables to examine the influencing factors that affect health facilities for the delivery of care. For all models, fixed effects were presented as odds ratios and 95% confidence intervals. Akaike's information criterion (AIC) was used to measure the model fit. When the values of AIC remain lower, it indicates that the model fits better than the former model. Many researchers have identified multicollinearity as a high level of interdependence between independent variables. It would be a matter of concern if the tolerance value was 0.1 or less than that, and the cut-off point of the variance inflation factor (VIF) of 5 or 10 was considered.

For data management and analysis, Microsoft Excel, the Statistical Package for Social Sciences (SPSS) version 25, and R version 4.0.0 software were used. The SUMMER package [30] is used to show geographical trends.

### 2.5. Ethical Statement

The study used publicly available data from the Multiple Indicator Cluster Survey (https://mics.unicef.org/), and the shape file was downloaded from the Humanitarian Data Exchange (https://data.humdata.org/), which was open to all. As a result, no additional ethical approval is required for this investigation.

## 3. Results

### 3.1. Trends of Health Facility Delivery in Bangladesh

In addition to the data from the Bangladesh Multiple Indicator Cluster survey for 2019, we also used the data from the Bangladesh Multiple Indicator Cluster Surveys for 2006 and 2012-13 in this study to show the trend of the delivery of health facilities in Bangladesh (Figures 2 and 3).

The trend of using health facilities during delivery from 2006 to 2019 in Bangladesh is shown in Figure 2. This trend showed an increasing rate of using health facilities during delivery from 16% to 53.4% over the years. The geographical illustration of the health facilities during delivery over the years is expressed in Figure 3. Here, Bangladesh was divided into three distinct territories according to the use of health facilities in delivery in 2006, 2012-13, and 2019 red, orange, and green. From the geographical illustration, in 2006, the maximum districts of Bangladesh had a lower percentage of women who used health facilities during delivery (the red color shows the lower percentage). However, this rate was gradually increasing over time, and the rate of using healthcare facilities during delivery was higher in 2019 which is shown in green.

### 3.2. Background Characteristics of Cofactors

In this study, we included 7,950 and 9,183 women, aged 15 to 49 years, from 2012-13 and 2019, who had given birth live in the past two years. In Table 1, we show the proportion of women based on factors at the individual and community levels.

The highest percentage of women across the study period was 20-34 years. Approximately 31.6% of women had preprimary or no formal education in 2012-13. Half of the 9183 women completed their secondary education, and about 9% of the women had preschool education or no education in 2019. Most women (above 91%) in our country belong to Islam. About 43.2% of women were poor in 2012-13. Women's economic status increased from 37.6% in 2012-13 to 40.9% in 2019. More than half (53.3%) of the women had 2-3 children and 75.1% wanted children in 2019. The results showed that approximately 78% of the women lived in rural areas in each sample. About 31.5% and 7.9% of women lived in the Dhaka and Sylhet divisions, respectively, in 2012-13 which was 24.1% and 8.4% in 2019. The percentage of women from other divisions was almost the same over the periods. Women with exposure to the media had a better rate (60.6%) than those without exposure (39.4%) in 2019. Approximately 41.0% of women reported 1-3 times of prenatal care during their pregnancy in 2012-13, which increased by 45.9% in 2019. Finally, women who provided skilled prenatal care during pregnancy were 71.7% in 2019, whereas the percentage was 58.3% in 2012-13.

### 3.3. Bivariate Analysis

In Table 2, the results showed significant relationships between the use of health facility delivery with the individual and community-level characteristics of women. The use of health facility delivery was higher among women aged 20-34 years, which was 54.7% in 2019. About 80.6% of women with higher and above education received healthcare facilities during delivery in 2019, which was 66.6% in 2012-13. The results showed that 30.0% of women who received facilities during delivery were from Islam, which increased by 52.3% in 2019. Approximately 65.9% of women of other religions were more likely to use health facilities than Muslims in 2019. In the socioeconomic context, a large portion (73%) of women from richer families received health facility delivery services compared to women from middle class or poorer families in 2019. Approximately 28.2% of women who had 2-3 living children received health facility delivery in 2012-13 which increased by 50.8% in 2019.

The prevalence of health facilities during delivery of women had increased from 49.9% in 2012-13 to 67.7% in 2019 in urban areas. About 34.9% of women from the Dhaka division received health facility delivery in 2012-13, which later increased by 62.0% in 2019. The highest percentage of women received facilities in delivery from the Khulna division. Approximately 63.9% of women who were exposed to the media used health facilities during delivery in 2019. Women who reported three or more prenatal visits had a higher rate of delivery at the health facility than women who reported one prenatal visit. The study found that a large portion (64.8%) of facilitated women obtained skilled prenatal care providers during delivery in 2019.

### 3.4. Collinearity Diagnostic

Table 3 illustrates when the interdependence among independent variables is at a high level, which is defined as multicollinearity. In a regression model, the presence of multicollinearity might reduce the precision of estimation, which would be difficult for studies. For this reason, we examined the multicollinearity among independent variables in Table 3. In terms of the cut-off point of the variance inflation factor (VIF) and tolerance [31], we discovered that all values covered the tolerance range of tolerance (>0.1) and the VIF value (<2.5). We concluded that there was no multicollinearity occurring in this study.

### 3.5. Measures of Fixed and Random Effects

The results of the random intercept multilevel logistic regression with two-level factors are three models, including one unconditional or empty model and two conditional models. The effects of explanatory factors on health facility delivery status are presented in Table 4. Here, we fit two different two-level logistic regression models, one for Bangladesh MICS, 2012-13 (model 1A, model 2A, and model 3A), and another for Bangladesh MICS, 2019 (model 1B, model 2B, and model 3B).

### 3.6. Unconditional or Null Model (Models 1A and 1B)

This study first proposed an intercept-only model to evaluate whether our data justified the decision to estimate random effects at the cluster level. As shown in models 1A and 1B (empty model) in Table 4, there were significant differences in the possibility of delivery across clusters or communities in medical institutions. The estimated variation in the delivery of health care explained by model 1B (that is, the year 2019) is 1.13 at the community level, which was reduced from the 2012-13 estimate (1.25 for model 1A). The percentage of intraclass correlation (ICC) in the intercept-only model is 26% in 2019, which indicates that there exists about 26% of heterogeneity between the two individual- and community-level factors and a two-level regression model can be applied in this study. In the 2012-13 estimate, this percentage was 28%.

### 3.7. Individual-Level Model (Models 2A and 2B)

In this model, we include only individual-level covariates as fixed effects, that is, the age of the women in years, the educational level of the women, the status of household wealth, religion, the wanted children, and the children ever born.

According to model 2 (both 2A and 2B) in Table 4, the age of women showed a significant and positive association with the use of health care delivery services. Here, the use of healthcare delivery has increased among younger women compared to older women over the years but is lower among younger women than older women for both surveys. For example, women aged 15 to 19 years used 30% (OR = 0.70, 95% CI: 0.54-0.91) fewer healthy facilities during delivery in 2019 compared to women aged 35 to 49 years; the percentage was 34% less (OR = 0.66, 95% CI: 0.48-0.91) in 2012-13. That is, it can be concluded that there was an improvement in the trend of maternal age to use health facilities for delivery in Bangladesh.

Women's education showed a significant and positive relationship with health facility delivery. The results demonstrated that women who had fewer educational qualifications used fewer healthy facilities during their delivery period than highly educated women. In this case, the odds ratio increased among women with secondary education from 0.46 in 2012-13 to 0.52 in 2019. In terms of preprimary/no education, the odds ratio shows a negative trend from 2012-13 to 2019-time frame (OR (2012 − 13) = 0.21, 95% CI: 0.17-0.26 and OR (2019) = 0.18, 95% CI: 0.14-0.23).

Findings from model 2 also showed that the possibility of using a health facility during delivery increased with increases in household wealth status. That is, the lower the family status, the less the facility is used. For example, women in poor and middle-class families were 75% (OR = 0.25, 95% CI: 0.22-0.28) and 53% (OR = 0.47, 95% CI: 0.40-0.54) less likely to use healthy facilities during delivery than women in rich families in 2019.

The rates of use of health facilities' delivery services were lower in Muslim families than in others, although this rate decreased by 24% (OR = 0.79 in 2012-13 and OR = 0.55 in 2019). The probability of giving birth in a medical institution decreases as the number of children born ever increases over the years. For example, the odds were 2.45 for one live births and 1.49 for 2-3 live births in 2019. The estimated community-level variance in models 2A and 2B is 0.65 and 0.54, respectively, and the ICC is 17% and 14%.

### 3.8. Individual- and Community-Level Model (Models 3A and 3B)

In model 3 (both 3A and 3B), after adding community-level factors, it is observed that individual-level factors consistently influence health facility delivery. At the same time, this model also demonstrates that women's education and the index of household wealth remain potential predictors of the delivery of health facilities. As in the previous model, lower education and economic levels indicate less use of health services during the delivery period.

The results of models 3A and 3B show that women residing in Dhaka (OR = 1.69, 95% CI: 1.28-2.22), Khulna (OR = 3.11, 95% CI: 2.31-4.18), and Rajshahi (OR = 2.48, 95% CI: 1.80-3.41) divisions had significantly higher usage of health facility delivery services compared to women residing in the Sylhet Division in 2012-13 but the odds decreased later. Women use fewer health facilities for delivery in Mymensingh division (OR = 0.71, 95% CI: 0.52-0.96) in 2019.

In terms of exposure to the media, it has been observed that women who had been in contact with the media were more likely to receive healthcare facilities than women who had not been in contact with the media. For example, the odds of receiving healthcare facilities were 19% (OR = 1.19, 95% CI: 1.03-1.38) in 2012-13 which increased to 38% (OR = 1.38, 95% CI: 1.23-1.55) in 2019. For women who do not receive prenatal care and a qualified birth attendant, naturally, their delivery services are less healthy than those who received them. Furthermore, after adjusting for community-level factors, the total variance for the delivery of health facilities for models 3A and 3B is 0.42 and 0.33, respectively, and the ICC is 11% and 9%.

## 4. Discussion

In this study, we have tried to examine the relationship between health facility delivery services and individual and community factors from the 2012-13 and 2019 Multiple Indicator Cluster Surveys in Bangladesh. The results show that half of all live births in the last two years have been delivered in a healthy environment and through a medical institution. During the past few decades, Bangladesh has made significant progress in reducing maternal and infant mortality and improving the reproductive health of women to achieve Millennium Development Goals (MDGs) 4 and 5 [32]. From the geographical illustration, we can say that the rate of receiving health facilities during the delivery period in 2019 is much higher than in 2006. However, this increase is not appropriate for Bangladesh, because the maternal mortality rate is still high in Bangladesh and the main reason is the lack of health facilities [33]. Bangladesh is a developing country with many health facility problems and has the lowest effective coverage [12, 33]. Not only Bangladesh but also many developing countries, such as Zambia and Tanzania, have the lowest level of healthcare delivery service [34, 35]. However, Ethiopia's healthy delivery rate is higher than that of Bangladesh [36].

In this study, individual factors are an important contributing factor to the delivery of health facilities over the years, especially, women's educational qualifications and family economic status. This study reveals that women's educational qualifications are the strongest predictor of health facility delivery in both periods of the MICS surveys (2012-13 and 2019). At the individual level, this study found that highly educated women were more likely to use health facilities during delivery and this rate increased during the study period. After all, the more educated women are, the more knowledge and awareness they can have about their health [37]. Therefore, educated women are more careful during pregnancy and delivery than less educated women. Researchers from different countries, including Bangladesh, expressed similar views on this study [38–43].

In terms of socioeconomic status, women who come from poor families or whose family financial status is poor try to use fewer health facilities during delivery in the 2012-13 and 2019 MICS surveys. This finding was in line with other studies which revealed that mothers who were in the richest households were less likely to have home deliveries compared to women in the poorest households [44–48].

In this study, a relationship was found between healthy delivery and the age of the women. Younger women have less knowledge about their delivery of health care. Previous research suggested that older women are more aware of the availability and accessibility of these services [49, 50].

Muslim women were more likely to have a birth at home than women of other religions. Similar to the findings of this study, various studies have also shown that women in Muslim families give birth in unhealthy environments at home [51, 52]. One of the main reasons for this is the religious convention. Women with 2-3 children naturally give birth in a healthy environment.

Place of residence is also an important factor only for MICS 2012-13. From this analysis, we found that those women from the urban household were higher odds of health facilities during delivery than their counterparts. This finding is consistent with the previous study of Bangladesh [43]. Again, this study found a significant association with the region in which women who resided in the Khulna, Rajshahi, and Dhaka divisions received more health facilities during delivery than in other divisions. This finding is consistent with the previous study [16, 43]. In terms of exposure to the mass media, this study found that women less well-known in the media were more likely to deliver at home. Previous research also found a connection between media access and the choice of birthplace women who are not familiar with the media are more likely to deliver at home [43, 53].

The study also found an association between prenatal care and delivery in health facilities delivery for the last two surveys (MICSs 2012-13 and 2019). This study found that women who had more prenatal care visits were more likely to have a facility delivery, consistent with previous research [54, 55]. Health professionals can provide pregnancy care to assist in delivery in health facilities. Women who were seen by skilled personnel were twice as likely to deliver in a healthy environment. This result is similar to studies conducted in Africa and concludes that receiving more skilled prenatal care was associated with an increased likelihood of delivery from health facilities [56].

In this study, clusters were used as the primary sampling unit, as a community, which does not represent the actual community level. This is one of the drawbacks of our research. This study has not been able to use the Bangladesh MICS, 2006 dataset because some variables were missing or were not found. Due to our data limitations, this study did not consider some important factors, such as the distance to the nearest medical center, the financial cost of transportation to the medical center, and the cultural barriers to providing medical services to the medical center. Another limitation of our analysis is that cross-sectional studies do not permit a distinction between cause and effect.

Although there are some limitations to this study, it has presented maternity care in Bangladesh. For example, the analysis results show that the more PNC received by skilled providers, the more women are interested in health facilities. On the other hand, future research needs to reduce community variation by improving the mass media communication system, implementing more education projects for women, providing facilities within the reach of all classes, and so on.

## 5. Conclusions

Health is a basic human right. Regardless of age, gender, socioeconomic, or ethnic background, we believe that our health is our most basic and most important asset. Despite the increase in health awareness around the world, maternal mortality has not declined at all. It is still a big challenge for developing countries like Bangladesh. Both individual and community factors are responsible for health care in Bangladesh. Each factor plays a vital role in the decision-making of health care. The study found that women with higher education, good socioeconomic conditions, high media exposure, and adequate prenatal care usually have access to medical services. Bangladesh's evidence-based health policies and plans must be implemented under vigorous leadership. Therefore, we support decision-makers to improve women's quality of life through the appropriate use of health services. Appropriate measures to address these factors can significantly improve the delivery of health services.

## Figures and Tables

**Figure 1:** Study population and sample selection procedure for this study.

**Figure 2:** Trend of using health facilities during the delivery period in Bangladesh.

**Figure 3:** Geographical trends of health facility delivery in Bangladesh.

**Table 1:** Background characteristics of individual-level factors and community-level factors.

Variables	2012-13		2019	
	Frequency	Percentage	Frequency	Percentage
Individual-level factor				
Women's age (in year)				
° 15-19	929	11.7	1247	13.6
° 20-34	6244	78.5	7085	77.2
° 35-49	777	9.8	851	9.3
°Women's education				
° Preprimary/none	2516	31.6	842	9.2
° Primary	1231	15.5	2134	23.2
° Secondary	3043	38.3	4593	50.0
° Higher+	1160	14.6	1614	17.6
°Wealth status				
° Poor	3435	43.2	3682	40.1
° Middle	1524	19.2	1748	19.0
° Rich	2990	37.6	3754	40.9
°Religion				
° Islam	7287	91.6	8429	91.8
° Others	666	8.4	754	8.2
°Wanted children				
° Yes	6337	79.7	6897	75.1
° No	1613	20.3	2286	24.9
°CEB				
° 1	2912	36.6	3191	34.7
° 2-3	3857	48.5	4927	53.7
° >3	1180	14.8	1065	11.6
Community-level factors				
°Residence				
° Urban	1681	21.1	2013	21.9
° Rural	6268	78.9	7170	78.1
°Division				
° Barishal	475	6.0	508	5.5
° Chattogram	1851	23.3	1985	21.6
° Dhaka	2503	31.5	2218	24.1
° Khulna	760	9.6	929	10.1
° Mymensingh	—	—	710	7.7
° Rajshahi	850	10.7	1071	11.7
° Rangpur	886	11.1	996	10.8
° Sylhet	625	7.9	767	8.4
°Mass media exposure				
° Exposure	1883	23.7	5561	60.6
° Not exposure	6067	76.3	3622	39.4
°Prenatal care				
° None	2674	33.6	1579	17.2
° 1-3	3257	41.0	4211	45.9
° >3	2019	25.4	3392	36.9
°Skilled prenatal care provider				
° Yes	4637	58.3	6583	71.7
° No	3313	41.7	2600	28.3

CEB = child ever born.

**Table 2:** Association between cofactors and the delivery of health facilities in Bangladesh.

	Healthcare facility delivery					
	2012-13			2019		
Variables	Yes (%)	No (%)	*χ* ^2^ value (*p* value)	Yes (%)	No (%)	*χ* ^2^ value (*p* value)
Women's age (in year)						
15-19	33.3	66.7	46.46 (<0.001)	54.2	45.8	55.33 (<0.001)
20-34	32.0	68.0		54.7	45.3	
35-49	20.3	79.7		41.3	58.7	
Women's education						
Preprimary/none	14.5	85.5	1092.17 (<0.001)	24.1	75.9	1067.94 (<0.001)
Primary	20.6	79.4		35.7	64.3	
Secondary	35.2	64.8		57.4	42.6	
Higher+	66.6	33.4		80.6	19.4	
Wealth status						
Poor	15.1	84.9	1114.44 (<0.001)	33.2	66.8	1184.26 (<0.001)
Middle	23.7	76.3		53.8	46.2	
Rich	52.9	47.1		73.0	27.0	
Religion						
Islam	30.0	70.0	34.25 (<0.001)	52.3	47.7	51.68 (<0.001)
Others	41.0	59.0		65.9	34.1	
Wanted children						
Yes	31.1	67.9	20.10 (<0.001)	55.7	44.3	61.18 (<0.001)
No	26.3	73.7		46.3	53.7	
CEB						
1	41.2	58.8	301.04 (<0.001)	64.7	35.3	376.27 (<0.001)
2-3	28.2	71.8		50.8	49.2	
>3	14.8	75.2		31.8	68.2	
Community-level factors						
°Residence						
° Urban	49.9	50.1	355.94 (<0.001)	67.7	32.3	211.61 (<0.001)
° Rural	25.9	74.1		49.4	50.6	
°Division						
° Barishal	17.1	82.9	227.71 (<0.001)	37.4	62.6	416.78 (<0.001)
° Chattogram	27.1	72.9		51.7	48.3	
° Dhaka	34.9	65.1		62.0	38.0	
° Khulna	45.7	54.3		71.1	28.9	
° Mymensingh	—	—		33.5	66.5	
° Rajshahi	38.0	62.0		57.1	42.9	
° Rangpur	23.0	77.0		49.5	50.5	
° Sylhet	20.8	79.2		40.2	59.8	
°Mass media exposure						
° Exposure	38.9	61.1	72.63 (<0.001)	63.9	36.1	630.99 (<0.001)
° Not exposure	28.5	71.5		37.2	62.8	
°Prenatal care						
° None	8.2	91.8	1440.44 (<0.001)	19.3	80.7	1478.98 (<0.001)
° 1-3	31.8	68.2		48.1	51.9	
° >3	59.9	40.1		75.9	24.1	
°Skilled prenatal care provider						
° Yes	45.7	54.3	1138.00 (<0.001)	64.8	35.2	1207.88 (<0.001)
° No	10.3	89.7		24.6	75.4	

CEB = child ever born.

**Table 3:** Multicollinearity diagnosis among explanatory variables.

Variables	2012-13		2019	
	Tolerance	VIF	Tolerance	VIF
Women's age (in year)	0.641	1.56	0.707	1.42
Women's education	0.713	1.40	0.734	1.36
Wealth status	0.918	1.09	0.600	1.67
Religion	0.618	1.62	0.990	1.01
Wanted children	0.458	2.18	0.945	1.06
CEB	0.472	2.12	0.621	1.61
Residence	0.969	1.03	0.849	1.18
Division	0.987	1.01	0.963	1.04
Mass media exposure	0.662	1.51	0.780	1.28
Prenatal care	0.965	1.04	0.593	1.69
Skilled prenatal care provider	0.869	1.51	0.611	1.64

CEB = child ever born; VIF = variance inflation factor.

**Table 4:** Multilevel modeling of health facility delivery among women in Bangladesh over the years.

Variables	2012-13						2019					
	Model 1A		Model 2A		Model 3A		Model 1B		Model 2B		Model 3B	
	OR	CI	OR	CI	OR	CI	OR	CI	OR	CI	OR	CI
Fixed effect												
*Individual-level factors*												
Women's age (in year)												
15-19			0.66^∗^	0.48-0.91	0.63	0.45-0.87			0.70^∗∗^	0.54-0.91	0.74^∗^	0.57-0.97
20-34			0.78^∗^	0.61-1.01	0.74	0.58-0.96			0.90	0.74-1.10	0.97	0.79-1.19
35-49 (ref.)			1		1				1		1	
Women's education												
Preprimary/none			0.21^∗∗∗^	0.17-0.26	0.35^∗∗∗^	0.27-0.44			0.18^∗∗∗^	0.14-0.23	0.31^∗∗∗^	0.25-0.41
Primary			0.29^∗∗∗^	0.23-0.36	0.40^∗∗∗^	0.32-0.51			0.27^∗∗∗^	0.22-0.32	0.38^∗∗∗^	0.31-0.45
Secondary			0.46^∗∗∗^	0.38-0.55	0.55^∗∗∗^	0.45-0.66			0.52^∗∗∗^	0.45-0.61	0.60^∗∗∗^	0.51-0.70
Higher+ (ref.)			1		1				1		1	
Wealth status												
Poor			0.28^∗∗∗^	0.24-0.32	0.41^∗∗∗^	0.35-0.48			0.25^∗∗∗^	0.22-0.28	0.46^∗∗∗^	0.40-0.53
Middle			0.42^∗∗∗^	0.35-0.50	0.49^∗∗∗^	0.41-0.59			0.47^∗∗∗^	0.40-0.54	0.65^∗∗∗^	0.56-0.76
Rich (ref.)			1		1				1		1	
Religion												
Islam			0.79^∗^	0.65-0.97	0.71^∗∗^	0.57-0.87			0.55^∗∗∗^	0.46-0.66	0.52^∗∗∗^	0.43-0.63
Others (ref.)			1						1			
Wanted children												
Yes			0.98	0.83-1.15	0.97	0.82-1.14			1.05	0.93-1.18	1.06	0.94-1.20
No (ref.)			1		1				1		1	
CEB												
1			2.42^∗∗∗^	1.88-3.11	1.80^∗∗∗^	1.38-2.33			2.45^∗∗∗^	1.97-3.04	1.96^∗∗∗^	1.57-2.44
2-3			1.48^∗∗∗^	1.18-1.87	1.13	0.90-1.44			1.49^∗∗∗^	1.24-1.80	1.20	0.98-1.45
>3 (ref.)			1		1				1		1	
*Community-level factors*												
Residence												
Urban					1.43^∗∗∗^	1.19-1.71					1.15	0.99-1.34
Rural (ref.)					1						1	
Division												
Barisal					0.93	0.66-1.33					0.85	0.65-1.12
Chattogram					0.89	0.66-1.18					0.94	0.75-1.18
Dhaka					1.69^∗∗∗^	1.28-2.22					1.47^∗∗∗^	1.16-1.86
Khulna					3.11^∗∗∗^	2.31-4.18					2.69^∗∗∗^	2.08-3.46
Mymensingh					NA	NA					0.71^∗^	0.52-0.96
Rajshahi					2.48^∗∗∗^	1.80-3.41					1.86^∗∗∗^	1.43-2.41
Rangpur					1.13	0.89-1.56					1.14	0.89-1.47
Sylhet (ref.)					1						1	
Mass media exposure												
Exposure					1.19^∗^	1.03-1.38					1.38^∗∗∗^	1.23-1.55
Not exposure (ref.)					1						1	
Prenatal care												
None					0.31^∗∗∗^	0.23-0.41					0.30^∗∗∗^	0.24-0.37
1-3					0.46^∗∗∗^	0.40-0.54					0.40^∗∗∗^	0.36-0.45
>3 (ref.)					1						1	
Skilled PNC provider												
Yes					2.68^∗∗∗^	2.10-3.42					2.31^∗∗∗^	1.96-2.71
No (ref.)					1						1	
Random effect												
Community-level variance	1.25		0.65		0.42		1.13		0.54		0.33	
AIC	9003.7		7888.9		7110.0		12414.8		10898.8		9935.3	
BIC	9017.6		7979.5		7277.2		12429.0		10991.5		10113.7	
Log likelihood	-4499.8		-3931.4		-3531.0		-6205.4		-5436.4		-4942.6	
Deviance	8999.7		7862.9		7062.0		12410.8		10872.8		9885.3	
ICC (%)	28.0		17.0		11.0		26.0		14.0		9.0	

Ref. = reference category; PNC = prenatal care. Statistical significance: ^∗^*p* < 0.05, ^∗∗^*p* < 0.01, and ^∗∗∗^*p* < 0.001.

## Data Availability

The study used publicly available data from the Multiple Indicator Cluster Survey (https://mics.unicef.org/) and the shape file was downloaded from the Humanitarian data exchange (https://data.humdata.org/) which was open to all.
